# Hyaluronidase in Clinical Isolates of *Propionibacterium acnes*

**DOI:** 10.1155/2015/218918

**Published:** 2015-02-18

**Authors:** Harmony Tyner, Robin Patel

**Affiliations:** ^1^Division of Infectious Diseases, Department of Medicine, Mayo Clinic, Rochester, MN, USA; ^2^Division of Clinical Microbiology, Department of Laboratory Medicine and Pathology, Mayo Clinic, 200 First Street SW, Rochester, MN 55905, USA

## Abstract

*Objectives*. We sought to describe the prevalence of a hyaluronidase gene and hyaluronidase production in 197 clinical isolates of *P. acnes*; we assessed kinetics of hyaluronidase production in a subset of three isolates. *Methods*. The hyaluronidase gene was detected using polymerase chain reaction. Hyaluronidase production was detected by growing isolates on BHI agar containing 400 *μ*g/mL hyaluronic acid and 1% albumin and flooding plates with 2 N glacial acetic acid to precipitate unbound hyaluronic acid, with a zone of clearing representing a positive phenotype. Hyaluronidase production kinetics were measured as a function of hyaluronic acid digestion over time in a liquid medium. *Results*. A hyaluronidase gene and hyaluronidase production were detected in 100 and 97% of *P. acnes* isolates, respectively. Hyaluronidase production in liquid medium was detectable after 96 hours of growth. *Conclusions*. Hyaluronidase production is nearly universal among *P. acnes* isolates. Three days appear to be required for significant hyaluronidase production in a liquid medium. Detection of hyaluronidase in tissue specimens may be a strategy to differentiate *P. acnes* infection from colonization when *P. acnes* is isolated from a clinical specimen.

## 1. Introduction

A slow-growing member of the normal microbiota of sebaceous glands which may be beyond the reach of topical antiseptics,* Propionibacterium acnes,* has long been recognized as a contaminant in clinical cultures. In specific clinical scenarios, however,* P. acnes* is increasingly recognized as a pathogen. Notable examples include* P. acnes* shoulder arthroplasty- and spinal instrumentation-associated infection. Recognition of the pathogenicity of* P. acnes* in such cases is dependent on its recovery from multiple separately collected specimens from a site expected to be sterile, in association with clinical symptoms. Because* P. acnes* has traditionally been considered a contaminant, its recovery has not been historically emphasized in clinical microbiology laboratories. And despite its recognition as a pathogen, it is also frequently isolated as a contaminant. Recent studies have informed strategies for ideal recovery of pathogenic* P. acnes* from clinical specimens [1, 2], but this issue remains a topic of controversy.

The main symptom associated with* P. acnes* orthopedic foreign body infection is pain. Other findings classically associated with infection, including fever and elevated white blood count (WBC), sedimentation rate (ESR), and C-reactive protein (CRP), are uncommon. The absence of abnormal inflammatory markers and other typical signs of bacterial infection may lead to* P. acnes* infection being disregarded because, despite repeated isolation of this organism, other findings pointing to a diagnosis of implant-associated infection may be lacking. Current guidelines for prosthetic joint infection (PJI) diagnosis [3] rely on features that may be absent in* P. acnes* PJI.

The reason for the paucity of acute inflammatory markers associated with* P. acnes* infection remains incompletely defined.* P. acnes* secretes a number of proteins [4]; the* P. acnes* secretome includes 20 proteins. The identity and function of only a few of these proteins have been described and characterized. Among the proteins in the secretome are the enzymes hyaluronidase, chondroitin sulfatase, and gelatinase [5, 6]. Hyaluronidases are enzymes that degrade hyaluronic acid, a component of the extracellular matrix. Hyaluronic acid is present in tissues throughout the body, including bones and joints, contributing to the viscosity of synovial fluid and the lubrication of joints. It is also a part of the extracellular structure of chondrocytes involved in tissue healing. The ability of bacteria to degrade hyaluronic acid may be a virulence factor, enabling penetration of hyaluronidase-producing organisms into tissues rich in hyaluronic acid, including joints, creating an advantage for establishing growth in articular spaces. In addition to* P. acnes*, other Gram-positive pathogens, such as* Streptococcus pneumoniae, Streptococcus intermedius*,* Streptococcus constellatus*,* Streptococcus dysgalactiae, Staphylococcus aureus, Peptostreptococcus* species,* Clostridium perfringens*, and* Clostridium septicum*, as well as other species of* Propionibacterium*, including* P. granulosum*, produce hyaluronidase [7].

Herein, we defined the prevalence of a hyaluronidase gene and of hyaluronidase production in a collection of clinical isolates of* P. acnes*. We also defined the time course of* in vitro* hyaluronidase production by* P. acnes* using a subset of three clinical isolates.

## 2. Methods

### 2.1. *P. acnes *Isolate Collection

197 clinical isolates of* P. acnes* were studied, including isolates associated with clinically significant monomicrobial infections, such as PJI, spine infections, and endocarditis, as well as isolates from clinical specimens with polymicrobial growth and isolates representing contamination (Table 1). Of the 197 isolates, 71 were associated with clinically significant growth, defined as growth of ≥20 colony forming units/10 mL sonicate fluid [8] or ≥3 positive cultures. All 197 isolates underwent molecular testing for a* P. acnes* hyaluronidase gene and phenotypic testing for hyaluronidase production; three isolates underwent time-course studies for assessment of kinetics of hyaluronidase production.

### 2.2. Genotypic Detection of Hyaluronidase Gene

*P. acnes* isolates were grown under anaerobic conditions in 2 mL brain heart infusion broth supplemented with 1% glucose, with agitation. DNA was extracted using the QIAamp UCP Pathogen Mini Kit (QIAGEN, Valencia, CA) with a final elution into 50 *μ*L elution buffer. A 451-base-pair region of the hyaluronidase gene sequence [9] was targeted by polymerase chain reaction (PCR) primers, forward primer 5′-TTTCGGGATCCTTGTGGTA-3′, and reverse primer 5′-TCTGGACAACAAACCTGT-3′. Primer sequences were selected from the published* P. acnes* hyaluronidase gene sequence [9]. Basic Local Assignment Search Tool (BLAST) analysis showed that the primer sequences had complete matches only with the two published* P. acnes* hyaluronidase gene sequences. 5 *μ*L of isolated DNA was amplified using 42 cycles as follows: melting at 95°C for 30 seconds, annealing at 54°C for 60 seconds, and amplifying at 72°C for 120 seconds. The final product was run on a 1% agarose gel and the product identified based on amplified product size. Amplified DNA from a representative isolate was sequenced and the following sequence was obtained: ‘CGCCCGCCGTGTGCTGTAGGTCTTCGGGGCTGGGGTCAGGGTTGGTGCTGGTTGTTATGAAGGGCGAGTGCGCCTTGCGGGGGTCTGCCGAGATCAGAACGGTCTGACGGCTCGAGCCGGATACGAGGTCGGTGAGGATCTCGGCGACCTTCCGGTCGGTCTTGGCGATGATCGCTCGGGCACGTGGGTCAGAGGTCCGGGCGGCTCTGCGTCCGGTGATGATGTCGATCCATCGCTCGCACAGCGCCGACCAGCTGTCGGGCCCGGGGGCGGCAATGGCGTCCGTCACTGTGGGAGAAGCGGCGAGCGCCATGGCTGACAGCGCAGATGCGGTGAGGAAGGTTCGTCGAGATGGGGTGCCGAACAAGGGTCACGCTCCTCGGGAGAGGGTGGCAGCACTGCCACACGTACAGGTTTGTTGTCCAGA-3′, consistent with the* P. acnes* hyaluronidase gene.

### 2.3. Phenotypic Detection of Hyaluronidase Production

Hyaluronidase production was evaluated as described by Smith and Willett [5] and used as a binary determinant of the ability of each isolate to produce hyaluronic acid. Briefly, 100 mL brain heart infusion media was prepared with 1 g of agar, autoclaved at 121°C for 15 min, and cooled to 46°C; then, a 2 mg/mL solution of sodium hyaluronidase, boiled for 10 minutes to achieve solubility, was added to the cooled medium to a final concentration of 400 *μ*g/mL. 5% bovine albumin fraction *V* was added under constant stirring to yield a final concentration of 1%. Plates were poured to a depth of 3-4 mm and allowed to solidify at 4°C.* P. acnes* isolates were grown on sheep blood agar under anaerobic conditions until growth was observed. A single colony was streaked onto the hyaluronic acid medium, incubated under anaerobic conditions, and observed daily until growth was observed (24 to 72 hours). On the day growth was first observed, the plate was flooded with 2 N glacial acetic acid, which binds hyaluronic acid and albumin forming a white precipitate. Hyaluronidase production was considered to have been present if a zone of clearing was observed.

### 2.4. Time Course Studies of Hyaluronidase Production

The method was modified from that described by Tolksdorf and McCready [10]. The assay measures turbidity resulting from hyaluronic acid mixed with albumin in an acidic solution; hyaluronidase activity is measured as lack of turbidity. Standard curves of hyaluronic acid turbidity and hyaluronidase activity were constructed. Hyaluronic acid sodium salt from* Streptococcus equi* (Sigma, St. Louis, MO) was used for constructing the standard curve and for experimental readings, and hyaluronidase from bovine testes (Sigma) was used to define a standard curve of enzyme concentration/activity (Figures 1(a) and 1(b)). Based on these standardized curves, the limit of detection was 0.0125 *μ*g/*μ*L hyaluronidase, and the assay was fully saturated at 0.05 *μ*g/*μ*L hyaluronidase (Figure 1(b)).

To quantify production of hyaluronidase over time, three clinical isolates of* P. acnes* were grown anaerobically on sheep blood agar for two days. One was selected based on its lack of production of hyaluronidase using the plate method. The other two produced hyaluronidase, as determined using the plate method, one of which was observed to grow quickly (IDRL-7844) and the other of which took longer than 48 hours to exhibit visible growth (IDRL-7751). The isolates were suspended in brain heart infusion broth supplemented with 1% glucose to a turbidity of 1.0 McFarland and diluted 1 : 50 with glucose-supplemented brain heart infusion broth. 200 *μ*L was inoculated in triplicate in a 96-well tissue culture plate, with 7 identical plates prepared in duplicate. One half of the plates was incubated anaerobically using AnaeroPack System (Mitsubishi Gas Chemical America, Inc., New York, NY), and one half was incubated aerobically. At 6, 12, 24, 48, 72, 96, 120, and 144 hours, a single plate was removed from each incubator, the OD_600_ documented to assess planktonic growth, and the supernatant broth collected and filtered using a 0.2 *μ*m membrane filter to abort further enzyme production by removing viable bacteria and prevent turbidity of bacterial growth from influencing the OD_540_ reading done to detect enzyme activity based on precipitation. 85 *μ*L of a 0.4 mg/mL solution of hyaluronic acid was combined with 85 *μ*L of sample broth supernatant and allowed to react at 37°C for 10 minutes. The samples were then treated with 135 *μ*L of an acidic albumin reagent described by Tolksdorf and McCready made of 2.5 g bovine serum albumin, fraction *V* in 1000 mL of 0.5 M sodium acetate buffer at pH 4.2, for 10 minutes, following which the OD_540_ was measured (Figure 2) [10].

## 3. Results

### 3.1. Genotypic Detection of Hyaluronidase Gene

Of the 197 clinical isolates evaluated, all (100%) were positive for hyaluronidase gene (Figure 3).

### 3.2. Phenotypic Detection of Hyaluronidase Production

Of the 197 isolates tested, 191 (97%) produced hyaluronidase, characterized by a zone of clearing around colonies (Figure 4). The clinical isolates of* P. acnes* showed some variation in time to achieve robust bacterial growth. Most achieved detectable plate growth by 24 hours; however, some took as long as 72 hours of incubation before detectable plate growth was observed.

### 3.3. Time Course Studies of Hyaluronidase Production

When the two hyaluronidase-producing* P. acnes* isolates were grown anaerobically, hyaluronidase was detectable in solution by 96 hours and continued to accumulate over time (Figure 2), suggesting that hyaluronidase production begins when the organism reaches logarithmic phase growth. Hyaluronidase production did not occur under aerobic conditions (Figure 5).

## 4. Discussion

Hyaluronic acid is a component of skin and extracellular matrix found throughout the body, primarily in soft tissue. Hyaluronidase is the term used to describe any enzyme able to cleave hyaluronic acid. There are several distinct hyaluronidases including enzymes found in mammalian spermatozoa, in the saliva of parasites, such as leeches, and in bacteria. Bacterial hyaluronidases are similar to one another in that the end product of bacterial hyaluronidases is unsaturated disaccharides. This is distinct from mammalian and parasitic hyaluronidases [7]. A variety of Gram-positive human pathogens excrete hyaluronidase, an enzyme that may enable bacterial spreading and tissue penetration [7]. These include species of* Streptococcus*,* Staphylococcus, Peptostreptococcus*, and* Clostridium* listed previously, in addition to* P. acnes*. Gram-negative bacteria may also produce hyaluronidase; however, rather than excreting the enzyme extracellularly, the hyaluronidase they produce is a periplasmic enzyme and as such is less likely to aid in tissue penetration than is the enzyme produced by Gram-positive bacteria. Approximately 50% of the hyaluronic acid in the human body is found in the skin, though it is rich in articular spaces as well. As such, organisms able to cleave hyaluronic acid may be favored as agents of infection in these locations, aided by their enhanced ability to penetrate these spaces.

Results of our investigation show that all tested clinical isolates of* P. acnes* have the described hyaluronidase gene, and most have the ability to cleave hyaluronic acid. Organisms that tested positive by PCR, but which were unable to cleave hyaluronic acid, may have mutations in the hyaluronidase gene or its regulators. The ubiquity of the amplified genetic sequence is noteworthy as it suggests that the hyaluronidase is important to the core genome of* P. acnes*. The widespread presence of this gene in* P. acnes* makes it appealing to consider it as a potential genetic target for detection of* P. acnes* in clinical specimens [11, 12].

The nearly universal phenotypic ability to cleave hyaluronic acid is notable not only as a potential functional virulence mechanism but also as a potential tool for determining whether* P. acnes* isolated from a clinical specimen is a contaminant or a pathogen; given the results of the time-course studies in liquid medium, the enzyme may only be present in clinical tissue specimens in true infections. In our experiments using liquid media, hyaluronidase production was detected by approximately 96 hours of anaerobic growth. This contrasted with the observed 24 to 72 hours it took for* P. acnes* to produce detectable quantities of hyaluronidase using the plate method. The reason for the difference in time to detectable hyaluronidase production may be attributable to the lower inoculum used in the studies in liquid compared to solid media. Alternatively, it may be a consequence of the density of growth, which would be higher sooner on plates than in liquid medium. In clinical specimens collected from discrete physiologic spaces from which* P. acnes* is isolated, the presence of hyaluronidase may, hypothetically, support the sustained presence and growth of* P. acnes* in that site, which would not be expected to be the case when the* P. acnes* isolated is a contaminant, since a newly introduced contaminant would not have had sufficient time to accumulate detectable quantities of hyaluronidase. This may provide a tool for differentiating between contamination and sustained growth, even if no living organism is isolated from a specimen. Of note, other organisms are known to produce hyaluronidase, though their requisite growth conditions for hyaluronidase production and kinetics thereof are outside the scope of this paper.

Demonstrating that an enzyme such as hyaluronidase can be detected as a byproduct of* P. acnes* growth is a novel potential approach to detecting and characterizing infections and could set precedent for using byproducts of growth as a means of differentiating between contamination and sustained growth of this organism and others in clinical specimens. Describing the secreted and excreted products associated with bacterial growth has potential diagnostic implications not only for* P. acnes* but also for many organisms. The* P. acnes* secretome has been described and 20 proteins have been identified, though not all have been characterized. Exactly how unique each organism's secretome is, is unknown; however, it is likely that the secretome varies from organism to organism and could potentially be used as a “fingerprint” of growth to signify specific organism-types in clinical specimens, even in the case of nonculturable organisms. Given a lack of information on the secretome of common pathogens, a discussion of the broader application of using secreted or excreted proteins for detecting and characterizing bacterial growth from clinical specimens remains academic, aside from the established use of urease production for diagnosing* Helicobacter pylori* infection. This may represent an approach to more broadly detect and characterize infection, particularly in cases where there is a question of potential contamination.

The environment of the articular space has been a subject of debate and the question has been raised over time as to what oxygen tension is present in the joint space. It has been suggested that articular spaces may have lower oxygen content than other locations in the body [13].* P. acnes* typically grows better under anaerobic than aerobic conditions. Our observation that* P. acnes* hyaluronidase is produced under anaerobic but not aerobic conditions (Figure 4) may have clinical relevance in the context of the environment in joint spaces and possibly in biofilms.

There are several limitations to our study. In cases where the gene segment of interest was present, but there was phenotypic negativity, we did not sequence the gene. Also, quantification of hyaluronidase production was performed on just three isolates. Further characterization of more isolates under a variety of conditions might be informative.

## 5. Conclusions

Most clinical isolates of* P. acnes* are capable of cleaving hyaluronic acid, and all tested clinical isolates of* P. acnes* had a hyaluronidase gene. The ubiquity of this characteristic in* P. acnes* isolates and the finding that the studied subset of isolates of* P. acnes* produced detectable quantities of hyaluronidase by 96 hours of sustained growth could hypothetically have diagnostic utility in differentiating between contamination with* P. acnes* and its presence as a pathogen in clinical specimens.* In vivo* and clinical studies would be useful to characterize the translation of our findings and to explore the use of excreted proteins in characterizing the significance of bacterial growth.

## Figures and Tables

**Figure 1:** (a) Standard curve used to measure hyaluronic acid concentration. Optical density of hyaluronic acid at 540 nanometers wavelength (OD_540_). (b) Standard curve used to measure hyaluronidase concentration. Hyaluronic acid will bind with albumin and form a white precipitate when acidified. When hyaluronidase is present, it digests hyaluronic acid, and the hyaluronic acid cannot bind with albumin and precipitate. Decreased precipitation is measured as increased light transmission and, therefore, a lower OD_540_ reading.

**Figure 2:** Kinetics of hyaluronidase production in* Propionibacterium acnes*. Three isolates were studied, including a hyaluronidase nonproducing (as determined by plate assay) isolate (*P. acnes* IDRL-7676) and two hyaluronidase-producing (as determined by plate assay) isolates (*P. acnes* IDRL-7751 and* P. acnes* IDRL-7844). Hyaluronidase production was measured by increased light transmission at OD_540_. Sterile medium was used as a negative control.

**Figure 3:** Genotypic detection of* P. acnes* hyaluronidase gene. Polymerase chain reaction assay was used to detect a 451-base-pair segment of the* P. acnes* hyaluronidase gene in 197* P. acnes* clinical isolates. This is a representative gel, demonstrating the appearance of a typical selection of isolates. The identity of each organism, by lane, is as follows: 1: IDRL-7421; 2: IDRL-7811; 3: IDRL-7812; 4: IDRL-8403; 5: IDRL-9037; 6: IDRL-6536; 7: IDRL-7599; 8: IDRL-7714; 9: IDRL-9038; 10: IDRL-7737.

**Figure 4:** Phenotypic detection of hyaluronidase production. Plates were prepared with brain heart infusion agar supplemented with hyaluronic acid and albumin.* P. acnes* isolates were allowed to grow until there was visible growth; thereafter, the plate was acidified with 2 N glacial acetic acid, causing undigested hyaluronic acid to bind to albumin, forming a white precipitate. Hyaluronidase production was considered to be present if a zone of clearing was observed.

**Figure 5:** Hyaluronidase production by* Propionibacterium acnes* under aerobic and anaerobic conditions. Two hyaluronidase-producing isolates of* P. acnes* were incubated under aerobic and anaerobic conditions. Hyaluronidase production was measured by light transmission at OD_540_. Hyaluronidase was detected with incubation under anaerobic but not aerobic conditions.

**Table 1:** Study isolates.

Source of isolation, number of isolates	% of all cases	Number with clinically significant growth (%)
Total number, 197	100%	71 (36%)
Upper extremity, including hardware and native joints, 36	18%	24 (67%)
Lower extremity, 51	26%	7 (14%)
Spine/vertebral hardware, 45	23%	25 (49%)
Breast implant, 49	25%	9 (18%)
Penile implant, 7	4%	1 (14%)
Cardiac valve, 3	2%	2 (67%)
Blood, 1	1%	1 (100%)
Pacemaker, 5	3%	2 (40%)

The table shows the site of isolation of the study isolates and whether they were considered to represent clinically significant growth (i.e., not contaminants).
